# Deep Learning-Based Computed Tomography Image Features in the Detection and Diagnosis of Perianal Abscess Tissue

**DOI:** 10.1155/2021/3706265

**Published:** 2021-08-03

**Authors:** Song Han, Jun Yang, Jihua Xu

**Affiliations:** Department of Anorectal Surgery, Qilu Hospital (Qingdao), Cheeloo College of Medicine, Shandong University, 758 Hefei Road, Qingdao 266035, Shandong, China

## Abstract

The performance characteristics of deep learning fully convolutional neural network (DLFCNN) algorithm-based computed tomography (CT) images were investigated in the detection and diagnosis of perianal abscess tissue. 60 patients who were medically diagnosed as perianal abscesses in the hospital were selected as the experimental group, and 60 healthy volunteers were selected as the control group. In this study, the DLFCNN algorithm based on deep learning was compared with the CNN algorithm and applied to the segmentation training of CT images of patients with perianal abscesses. Then, the segmentation metrics Jaccard, Dice coefficient, precision rate, and recall rate were compared by extracting the region of interest. The results showed that Jaccard (0.7326) calculated by the CNN algorithm was sharply lower than that of the DLFCNN algorithm (0.8525), and the Dice coefficient (0.7264) was also steeply lower than that of the DLFCNN algorithm (0.8434) (*P* < 0.05). The thickness range of the epidermis and dermis in patients from the experimental group was 4.1–4.9 mm, which was markedly greater than the range of the control group (1.8–3.6 mm) (*P* < 0.05). Besides, the CT value of the subcutaneous fascia in the experimental group (−95.45 ± 8.26) hugely reduced compared with the control group (−76.34 ± 7.69) (*P* < 0.05). The accuracy rate of the patients with perianal abscesses was 96.67% by multislice spiral CT (MSCT). Therefore, the DLFCNN algorithm in this study had good stability and good segmentation effect. The skin at the focal site of anal abscess was obviously thickened, and it was simple and accurate to use CT images in the diagnosis of patients with perianal abscesses, which could effectively locate the lesion and clarify the relationship between the lesion and the surrounding structure.

## 1. Introduction

Perianal region refers to the area extending 5-6 cm from the junction between the anal squamous mucosa and the skin [1]. Perianal abscess is an abscess caused by acute and chronic infections of the perianal space [2], which is manifested as redness, pain, swelling, and agglomeration of the skin around the anus, accompanied by systemic symptoms of varying degrees [3]. Perianal abscess is a common and frequently occurring disease in surgery, which has a high incidence and seriously affects the normal life and work of patients. In the past, the comprehensive diagnosis of perianal abscess was mainly made by digital surgical rectal examination, clinical symptoms, clinical vital signs, etc., which could not directly determine the location and range of the lesion and resulted in high blindness in diagnosis and treatment [4]. Therefore, the surgical treatment of perianal abscess has to be accurately positioned and diagnosed preoperatively to improve the safety of the surgery.

In recent years, with the continuous development of electronic imaging technology, multislice spiral computed tomography (MSCT) has gradually been applied in the clinical treatment of perianal abscess [5]. CT scanning has the characteristics of fast scanning speed, powerful image postprocessing function, and clear image [6]. Furthermore, CT scanning is used for the examination of the human abdomen and pelvis, without special bowel preparation such as enema or inflation [7]. Therefore, the application of CT scanning to examine the tissue structure of human perianal abscesses will help improve the clinical diagnosis of anal diseases.

Segmentation algorithms based on deep learning can deeply learn the mapping relationship between images and are widely used in computer vision and sound effects. They can methodically sort out a large amount of data, extract image features, and efficiently deal with complex problems, which have become the mainstream application of segmentation algorithms at present [8, 9]. Mastragostino et al. [10] used the deep learning-based convolutional neural network to evaluate CT images of liver tissue with high segmentation accuracy. In this study, a deep learning fully convolutional neural network (DLFCNN) algorithm was proposed to replace the full connection layer in the later stage of the CNN with the convolutional layer so that the number of neurons in the input layer was not restricted. The input of the convolutional layer could accept images of different sizes; the window for each value in the output to be mapped to the receptive field in the input image was fixed, which greatly improved the speed.

In this study, DLFCNN algorithm was proposed and compared with the CNN algorithm, which was applied in the CT imaging diagnosis of 60 patients with perianal abscesses. The objective of this study was to investigate the ability of CT images to distinguish the structure of perianal abscess tissue and to summarize the specific signs of perianal abscess tissue, so as to lay a foundation for the CT diagnosis of anorectal diseases.

## 2. Materials and Methods

### 2.1. General Data

In this study, 60 patients with medical diagnosis of perianal abscess in the Department of Anorectal Surgery of our hospital from October 2018 to December 2019 were selected as the experimental group, including 68 males and 52 females, with an average age of 54.23 ± 11.46 years. Another 60 healthy volunteers were selected as the control group, and the experimental group was diagnosed by MSCT scanning. The study was approved by the Medical Ethics Committee of the hospital, and the research objects and their family members learnt about the study and signed informed consent forms.

The criteria for inclusion were defined to include research objects who were diagnosed with perianal abscesses and had anal mass with pain, had complete clinical data and imaging data, and had suffered from the disease for more than 4 weeks.

The criteria for exclusion were defined to include research objects who were combined with cardiovascular disease, mental illness, speech impairment, and hearing impairment, did not undergo anorectal surgery in the past 6 months, and had unclear CT images.

### 2.2. Deep Learning Fully Convolutional Neural Network (DLFCNN) Algorithm

Neuron is the basic functional unit of the whole neural network structure (Figure 1). A large number of neurons together form a neural network structure. The essence of the internal convolution operation of the DLFCNN algorithm model is the integral operation, and the calculation equation is as follows:

(1) $$\begin{array}{c} \left(g\cdot h\right)\left(s\right)≜\int_{-\infty }^{\infty }g\left(\gamma \right)h\left(s-\gamma \right)\text{d}\gamma . \end{array}$$

In equation (1), function *g* and function *h* represent continuous functions, and both of them are integrable functions in the range of real numbers. Assume that the two-dimensional vector *P* and the convolution kernel *Q* are the input, and the output *L* is a two-dimensional tensor, which can be expressed in the following:

(2) $$\begin{array}{c} L\left(i,j\right)=\left(P\cdot Q\right)\left(i,j\right)=\sum_{a}\sum_{b}P\left(a+i,b+i\right)\cdot Q\left(a,b\right). \end{array}$$

In equation (2), *P* is a 6 × 6 two-dimensional vector, *Q* is a 4 × 4 convolution kernel, and the output *L* is a two-dimensional tensor with 4 × 4. According to the equation, the size of the input image (*i* × *i*) directly affects the size of the output image (*L* × *L*), and it will also be affected by the size of the convolution kernel (*q* × *q*) during the operation. In order to better segment the edge of the image, a supplementary parameter *o* is often added. The specific equation is as follows:

(3) $$\begin{array}{c} L=\left[\frac{i-q+2o}{t}\right]+1. \end{array}$$

In equation (3), *i* stands for the size of the input image, *q* represents the size of the convolution kernel, and *L* means the size of the output image. Model networks often have multilayer superimposed hollow convolution, and the use of a zigzag structure can avoid the superposition of information and maintain the continuity of information. The zigzag structure uses time intervals of different lengths to integrate information from different distances and nearby locations. Thus, the following equation can be obtained:

(4) $$\begin{array}{c} N_{i}=\text{max}\left[N_{i+1}-2\lambda_{i},N_{i+1}-2\left(N_{i+1}-\lambda_{i}\right),\lambda_{i}\right]. \end{array}$$

In equation (4), *λ*_*i*_ represents the hole interval of the *i*th layer, and *N*_*i*_ indicates the hole interval of the last layer, which is also the maximum value of the hole interval. In this study, the void interval was set to (2, 4, 5). The essence of the operation of the convolutional layer is to perform weighted summation. The function used in this study was the sigmoid function for classifying and outputting, and the ReLU function was adopted for extracting image features. Among them, the calculation and derivative equations of the sigmoid function are shown in the following:

(5) $$\begin{array}{c} \text{Sig}=\frac{1}{1+e^{-c}}=\frac{1}{1+e^{-\left(vx+b\right)}}, \end{array}$$

(6) $$\begin{array}{c} {\text{Sig}}^{\prime }\left(c\right)=\frac{e^{-c}}{{\left(1+e^{-c}\right)}^{2}}. \end{array}$$

The function values in equations (5) and (6) are both in (0, 1), and the sigmoid function is a differentiable function. The ReLU function can reduce the problem of the disappearance of the gradient, and its mathematical operation and derivative equations are as follows:

(7) $$\begin{array}{c} \text{ReLU}\left(c\right)=\text{max}\left(0,c\right), \end{array}$$

(8) $$\begin{array}{c} {\text{ReLU}}^{\prime }\left(c\right)=\left\{\begin{array}{c} 0,\;c<0,\\ 1,\;c>0. \end{array}\right) \end{array}$$

In equations (7) and (8), the derivative of the ReLU function is negative, and the gradient is in a saturated state when *c* < 0. When *c* > 0, the derivative of the ReLU function is 1, and no gradient disappears. Compared with the sigmoid function, the ReLU function has a faster calculation speed and convergence speed. For the input *P*, the gap between *g*(*P*) obtained by the model output and the actual value *K* usually requires a loss function to express the degree of deviation, which is recorded as *R*(*K*, *g*(*P*)) that is presented in the following equation:

(9) $$\begin{array}{c} R=\frac{1}{2m}\sum {\left(K-g\left(P\right)\right)}^{2}. \end{array}$$

### 2.3. Extraction of the Region of Interest from the CT Image of the Perianal Abscess Tissue

The main purpose of segmenting the CT image of the perianal abscess tissue was to classify the lesion. There was some irrelevant noise information in the CT image. If there was an error in the segmentation process, the classification result would be inaccurate, resulting in the perianal abscess. The iterative threshold method was adopted in this study to effectively solve the problems of inconspicuous contrast of light and dark in CT images, the dark overall image, and the too small difference between pixels. A clear CT image of perianal abscess could be obtained after a series of operations, such as expansion, corrosion, cavity filling, open operation, close operation, and mask operation.  Figure 2 shows the extraction process of the region of interest in the image of perianal abscess tissue through the iterative threshold method. After the extraction of the region of interest, the image of perianal abscess tissue could reduce the amount of data and the interference of noise, complete the outline of the lesion, and realize the preprocessing of the image.

### 2.4. Examination Method

The diagnosis was made by using Somatom Definition AS+ 64-slice, 128-slice 4-dimensional spiral CT (Siemens, Germany). Before the examination, routine bowel preparations were performed. After the bladder was properly filled, the scanning was started. Each patient held his head with his hands, his lower limbs were in an external stand, and he was in a supine position in the center of the examination bed. The central sagittal position of his body was perpendicular to the plane of the bed, and his head was advanced. During the examination, the patient should keep a calm state of mind, not move his body, and hold his breath as required.

Scanning parameters were as follows: the flat sweep tube voltage was 120 kV and tube current was 175 mA; layer thickness was 2.5 mm and layer spacing was 5.0 mm; enhanced tube voltage and tube current were also 120 kV and 175 mA in turn; scanning rotation speed was 0.8 s/r, pitch was 1.0, field of view (FOV) was 250 mm × 250 mm, and the matrix was 512 × 512; the reconstruction layer thickness was 1.5 mm, and the layer spacing was 1.5 mm. 0.9% sodium chloride (NaCl) injection and 20 mL of iohexol injection were used as contrast agents. After probe exploration, the catheter was inserted, and the contrast agent was injected. After completion, image processing was carried out. On the AmbiVU 4.2.3 workstation, the image of the third sacral vertebra-anus area was reconstructed with a thickness of 1.5 mm, and the multiplanar reconstruction and maximum intensity projection reconstruction technology were employed to observe and save the relevant data. Two experienced doctors reviewed the CT images separately and reached a conclusion after discussion when their opinions were inconsistent.

### 2.5. Simulation Experiment Design of Deep Learning Fully Convolutional Neural Network Algorithm

In order to verify the effectiveness of the CT image segmentation method of perianal abscess tissue based on DLFCNN, a comparative experimental platform was designed in this study. The CT images of 60 patients with perianal abscesses were processed in batch by DLFCNN based on deep learning. Colloidal operation was performed in the convolutional layer of the convolutional network. Finally, the segmentation results were output in the output layer of the full connection layer.  Table 1 shows the number of feature graphs and the size of the convolution kernel in each convolutional layer of DLFCNN. Moreover, C1 represented the convolutional layer, which mainly performed the convolution operation of the filter and then output the activation function. S2 stood for the sampling layer, and the input data of the previous layer were processed by dimensionality reduction. C3 and S4 both expressed the network layers, C3 was similar to C1, and S4 was similar to S2, which indicated the second downsampling layer. C5 meant the convolutional layer, which had 28 feature maps; the size of the feature map was changed after processing. S6 represented the downsampling layer, and the principles of C7 and S8 were the same as before. In addition, F9 stood for the full connection layer, which contained multiple neural units, and each neural unit was fully connected to the previous layer.

### 2.6. Design of Evaluation Indicators for Deep Learning Fully Convolutional Neural Network Algorithm

In this study, it was necessary to select the appropriate image segmentation indicators in order to evaluate the extraction effect of the perianal abscess tissue segmentation process in the segmentation method. Commonly used segmentation metrics included Jaccard, Dice coefficient, precision rate, and recall rate. Jaccard was mainly employed to evaluate the effect of image segmentation, which could be calculated as follows:

(10) $$\begin{array}{c} \text{Jaccard}=\frac{C\cap D}{C\cup D}. \end{array}$$

In equation (10), *C* stood for the label of the anal abscess tissue delineated in the image segmentation, representing the gold standard; *D* meant the segmentation result. If Jaccard = 1, the segmentation result completely overlapped with the gold standard. The Dice coefficient could be adopted to evaluate the similarity of two sets, and its equation is expressed as follows:

(11) $$\begin{array}{c} \text{Dice}=\frac{2\left|C\cap D\right|}{\left|C\right|+\left|D\right|}. \end{array}$$

In equation (11), Dice = 1 indicated that the segmentation result was very ideal. Besides, the calculation of accuracy was as follows:

(12) $$\begin{array}{c} \text{Accuracy rate}=\frac{\text{TP}}{\text{TP}+\text{FP}}. \end{array}$$

In equation (12), TP stood for that the detected perianal abscess tissue showed a true positive, and FP meant that the detected perianal abscess tissue showed a false positive. Furthermore, the equation for calculating the recall rate was as follows:

(13) $$\begin{array}{c} \text{RR}=\frac{\text{TP}}{\text{TP}+\text{FN}}. \end{array}$$

In equation (13), TP suggested that the detected perianal abscess tissue presented a true positive, and FN indicated that the detected perianal abscess tissue presented a false negative.

### 2.7. Statistical Methods

SPSS 22.0 statistical software was used for analysis. The data which met the normal distribution were represented by the mean ± standard deviation ($\bar{x}+s$), and the data of the nonnormal distribution were expressed as the frequency and percentage. Furthermore, the *t*-test or *χ*^2^ test was used for comparison between the control group and the experimental group. In addition, *P* < 0.05 indicated that the difference was statistically substantial.

## 3. Results

### 3.1. Comparison on CT Image Segmentation Effects of the Two Algorithms

Figure 3 shows the comparison of the CT image segmentation effect between the CNN and FCNN. In this study, the DLFCNN algorithm was proposed based on deep learning and compared with the CNN algorithm, which were applied in the CT image evaluation of 60 patients with perianal abscesses. According to the general structure, the segmentation effect of the CNN was not particularly prominent, while the segmentation of the DLFCNN was relatively accurate.

### 3.2. Analysis on the Simulation Effects of the Two Algorithms

The simulation effects of the two algorithms were compared, and the results are shown in Figure 4. The maximum entropy method of the DLFCNN algorithm in this study began to converge around 25 iterations. The final loss value of the CNN was around 0.09. The image segmentation algorithm of the algorithm explored in this study had a faster convergence rate than the CNN in the training process, and the lowest final loss value was between 0.03 and 0.04.

Jaccard (0.7326) calculated by the CNN algorithm was sharply lower than that of the DLFCNN algorithm (0.8525) (*P* < 0.05), and the Dice coefficient (0.7264) hugely dropped in contrast to that of the DLFCNN algorithm (0.8434) (*P* < 0.05). The precision rate and recall rate of the CNN were also lower than the rates of the FCNN, but there was no significant difference. It revealed that the CNN was prone to oversegmentation and missing-segmentation. If the gold standard was taken as a reference, it indicated that the segmentation results differed greatly between the gold standards. However, the segmentation indicators of the DLFCNN in this study were improved to varying degrees, and the segmentation effect was better than that of the CNN.

### 3.3. Comparison on the General Data of Research Objects from the Two Groups

There was a comparison on the general data of research objects from the two groups, as shown in Figure 5. There were 36 males (60%) and 24 females (40%) in the experimental group, while there were 32 males (53.33%) and 28 females (46.67%) in the control group. Thus, the gender ratio of the two groups had no obvious difference (*P* > 0.05). The age range of the experimental group was 42–65 years, and the age range of the control group was 45–67 years. There was no marked difference in age between the experimental group and the control group (*P* > 0.05).

### 3.4. CT Imaging Features of Patients with Perianal Abscesses

Figures 6 and 7 display the axial and coronal CT images of two cases with perianal abscesses, respectively. The CT image of the soft tissue around the anal canal showed U-shaped thickening, uneven density, low-density shadows in the center, blurred edges of the lesion, and obvious enhancement of the central lesion on the enhanced scan. The central low-density shadow showed no obvious enhancement. The short strips were clearly intensified and connected with the posterior edge of the anal canal.

### 3.5. The Thickness of the Epidermis and Dermis in the Research Objects from the Experimental Group and the Control Group

According to the statistical results, it was found that the thickness of the epidermis and dermis of men was 2.8–3.6 mm, and the thickness of the epidermis and dermis of women was 1.8–2.6 mm. The thickness of the epidermis and dermis of men was obviously greater than the thickness of women, and the difference was statistically significant (*P* < 0.05) (Figure 8); the thickness of the epidermis and dermis of the experimental group was 4.1–4.9 mm, and the thickness of the control group was 1.8–3.6 mm, so the thickness of the experimental group markedly increased compared with that of the control group (*P* < 0.05) (Figure 9).

### 3.6. Comparison on the CT Observation of the Superficial Fascia and Subcutaneous Fascia between the Experimental Group and the Control Group

The comparison results of the CT observation of the superficial fascia and subcutaneous fascia between the experimental group and the control group are presented in Figure 10. The display rate of the superficial fascia in the experimental group was 46.35%, and the display rate of the control group was 37.56%, so there was no marked difference between the two (*P* > 0.05). Furthermore, the CT value (−95.45 ± 8.26) of the subcutaneous fascia in patients from the experimental group was substantially greater than the value of the control group (−76.34 ± 7.69), with a statistical difference (*P* < 0.05).

### 3.7. The Detection Rate of CT Images in Patients with Perianal Abscesses

Figure 11 shows the accuracy and misdiagnosis rate of lesions in patients with perianal abscesses. 60 cases of perianal abscesses were examined by MSCT, 58 cases were in line with pathological examination, and 2 cases were misdiagnosed. After postoperative pathological examination, 58 patients had accurate location of the lesions, with an accuracy rate of 96.67%, including 21 cases of upper levator ani muscle abscess and 37 cases of lower levator ani muscle abscess.

## 4. Discussion

In this study, the deep learning fully convolutional neural network algorithm was compared with the CNN algorithm, which were applied to the segmentation training of CT images of patients with perianal abscesses to solve the problem that the segmentation effect was not ideal due to incomplete feature extraction of the CNN segmentation. By extracting the region of interest, the commonly applied segmentation metrics of medical images were compared, including Jaccard, Dice coefficient, accuracy, and recall rate [11]. The results disclosed that the maximum entropy method of the DLFCNN algorithm in this study started to converge when the times of iteration were around 25, and the final loss value of the CNN was around 0.09. The lowest loss value of the image segmentation algorithm in this study was between 0.03 and 0.04 in the final training, suggesting that the convergence speed of the DLFCNN was fast. Jaccard (0.7326) calculated by the CNN algorithm sharply reduced compared with the DLFCNN algorithm (0.8525); the Dice coefficient (0.7264) was obviously lower than the Dice coefficient (0.8434) of the DLFCNN algorithm (*P* < 0.05) [12]. It showed that the CNN was prone to oversegmentation and missing-segmentation. If the gold standard was used as a reference, it indicated that the segmentation results were quite different among the gold standards [13]. DLFCNN in this study was improved to varying degrees in terms of segmentation indicators, with good stability and good segmentation effects [14].

Perianal abscess is a common and frequently occurring disease after clinical surgery, which is generally caused by primary infection. Some perianal abscesses are caused by trauma, inflammatory lesions, and drug injection [15]. Under normal circumstances, clinical diagnosis focuses on the number of lesions and the location of the relationship between the lesion location and the levator ani muscle. Besides, the use of CT imaging diagnosis before surgery has a very positive significance in preventing postoperative recurrence. MSCT images continue to expand the diagnostic methods of perianal abscess tissue imaging. It has the characteristics of fast inspection, thin layers, and high resolution and is widely used in the diagnosis of anal diseases [16]. When perianal abscess is detected with MSCT, it is usually not affected by the weak peristalsis of the anorectum, with few motion artifacts, and the lesion can be clearly shown in the image. Perianal abscesses are affected by the pus, the boundaries are not clear, and the density of the abscess is not uniform over time. In this study, the CT value of the subcutaneous fascia of the experimental group was −95.45 ± 8.26, which was significantly lower than the value of the control group (−76.34 ± 7.69) (*P* < 0.05). It might be that patients with early perianal abscess had more inflammatory exudate, and the CT scan had a uniform density and a low CT value [17]. In the middle and late stages of the formation of pus in the perianal abscess tissue, the absorption or discharge of pus will occur, forming an abscess cavity, which is manifested as a thick wall and abscess cavity [18]. With enhanced CT scanning, it can be observed that the thick wall of the abscess is obviously strengthened, in a ring shape, and the abscess cavity is not strengthened, showing a lower density. After the CT image is segmented by the DLFCNN algorithm, the relationship between the perianal abscess and the anorectum can be better displayed, and the number and location of the abscess can be accurately located, providing a reliable basis for the treatment of clinicians [19]. 60 patients with perianal abscesses were examined by MSCT. 58 patients had accurate location of the lesion with an accuracy rate of 96.67%, which confirmed that the MSCT scan could clearly show the morphology and structure of the lesion, thereby providing intuitive clinical diagnosis. This was consistent with the research findings of Zhao et al. [20].

CT image measurement of skin thickness is mainly used in the application research of breast skin, but there are few reports on the research of skin thickness measurement in the anal area. The statistical results of this study found that the thickness of the epidermis and dermis of men was in the range of 2.8–3.6 mm, and the thickness of the epidermis and dermis of women was 1.8–2.6 mm. The thickness of the epidermis and dermis of men was markedly greater than that of women, and there was a statistically great difference (*P* < 0.05). Moreover, the thickness of the epidermis and dermis of the experimental group was 4.1–4.9 mm, and the thickness of the control group was 1.8–3.6 mm. The thickness of the epidermis and dermis of the experimental group was greatly larger than that of the control group (*P* < 0.05), meaning that the skin at the lesion site was significantly thickened when a lesion occurred in the anal area, which could clearly distinguish between perianal abscess and other anal diseases.

## 5. Conclusion

In this study, DLFCNN was compared with the CNN and applied to the CT images of 60 patients with perianal abscesses. The DLFCNN algorithm had good stability and segmentation effect, and the skin at the focal area of anal abscess was obviously thickened. The CT image was simple and accurate in the diagnosis of patients with perianal abscess, which could be applied to effectively locate the lesion and clarify the relationship between the lesion and the surrounding structure. The shortcomings of this study are that the sample size is small, and the DLFCNN training images are few. Subsequently, the sample size should be expanded to further improve the accuracy of image segmentation. In this study, MSCT was adopted to detect the perianal abscess tissue, which could improve the reference basis for the clinical development of the scientific surgical treatment plan, effectively reduce the incidence of lesion omission, and prevent the recurrence of the patient's disease.

## Figures and Tables

**Figure 1:** The basic structure of a neuron.

**Figure 2:** The extraction process of the region of interest in the image of perianal abscess tissue by the iterative threshold method.

**Figure 3:** Comparison on the segmentation effect of the two algorithms. (a) Input CT image of perianal abscess tissue. (b) Segmentation effect of CNN algorithm. (c) Segmentation effect of DLFCNN algorithm.

**Figure 4:** Comparison on simulation effects of the two algorithms. (a) Loss training curve diagram of the two algorithms. (b) Comparison of the segmentation indicators of the two algorithms; ^∗^meant *P* < 0.05 compared with the CNN.

**Figure 5:** Comparison on the general data of research objects from the two groups. (a) The proportion of gender between the experimental group and the control group. (b) The age distribution of the experimental group and the control group.

**Figure 6:** CT image with a perianal horseshoe abscess (asterisk) (case 1, a male patient, aged 53 years). (a) Axial CT image. (b) Coronal CT image.

**Figure 7:** CT image with the spread of abscess upward to the left levator ani muscle, forming an abscess (case 2, a male patient, aged 56 years). (a) Axial CT image. (b) Coronal CT image.

**Figure 8:** Comparison on dermal and epidermal thickness between men and women in the control group. ^∗^indicated *P* < 0.05 compared with men.

**Figure 9:** Comparison on epidermal and dermal thickness between the experimental group and the control group. ^∗^meant *P* < 0.05 compared with the experimental group.

**Figure 10:** Comparison on the CT observation of the superficial fascia and subcutaneous fascia between the experimental group and the control group. ^∗^indicated *P* < 0.05 in contrast to the experimental group.

**Figure 11:** The accuracy and misdiagnosis rate of lesions in patients with perianal abscesses.

**Table 1:** The number of feature maps of the DLFCNN and the size of the convolution kernel.

Convolutional layer	The number of feature maps	The size of the convolution kernel
C1	14	2 × 2
S2	14	5 × 5
C3	14	5 × 5
S4	14	2 × 2
C5	28	5 × 5
S6	28	2 × 2
C7	28	5 × 5
S8	28	2 × 2
F9	52	5 × 5

## Data Availability

No data were used to support this study.
